# Iptacopan Efficacy and Safety to Treat Paroxysmal Nocturnal Hemoglobinuria (PNH): A Systematic Review and Meta-Analysis

This article has been retracted.

**DOI:** 10.7759/cureus.67830

**Published:** 2024-08-26

**Authors:** Ibrahim M Dighriri, Reham M Al-Qahtani, Amal O Almutairi, Rahaf N Alhashbari, Hanin A Kanbeja, Salman A AlOjaimi, Mona A Aljuaid, Abdullah A Albaradi, Sahar T Almanjumi, Samah A Alqurashi, Maryam S Majrashi, Hatoon M Alansari, Ghayah A Jabbari, Abdulaziz S Alharbi, Amnah A Alnami

**Affiliations:** 1 Department of Pharmacy, King Abdulaziz Specialist Hospital, Taif, SAU; 2 College of Pharmacy, King Khalid University, Abha, SAU; 3 Department of Pharmacy, East Jeddah General Hospital, Jeddah, SAU; 4 Department of Pharmacy, Ibrand Pharmacy, Taif, SAU; 5 Department of Pharmacy, Polyclinic of Dr. Zaher Qadeeb Alban, Makkah, SAU; 6 Department of Pharmacy, Dr. Suliman Alhabib Medical Group, Khobar, SAU; 7 College of Pharmacy, Taif University, Taif, SAU; 8 Department of Pharmacy, Zahrat-Alrawdah Pharmacy, Buraydah, SAU; 9 Department of Pharmacy, United Pharmacy, Taif, SAU; 10 Department of Pharmacy, United Pharmacy, Makkah, SAU; 11 Department of Pharmacy, Ibrand Pharmacy, Jazan, SAU; 12 College of Pharmacy, Jazan University, Jazan, SAU; 13 College of Pharmacy, Umm AlQura University, Makkah, SAU; 14 Department of Pharmacy, Sabya General Hospital, Gazan, SAU

**Keywords:** lactate dehydrogenase, hemoglobin, hemolysis, complement inhibition, factor b inhibitor, iptacopan, paroxysmal nocturnal hemoglobinuria

## Abstract

Paroxysmal nocturnal hemoglobinuria (PNH) is an uncommon blood condition caused by complement-mediated hemolysis. In early clinical studies, iptacopan, an oral factor B inhibitor, showed promise in treating PNH. This systematic review aimed to compile information on the effectiveness and safety of iptacopan for PNH. A systematic review was performed using Preferred Reporting Items for Systematic Reviews and Meta-Analyses (PRISMA) standards. The Medline, Embase, PubMed, and Cochrane Central databases were searched for randomized controlled trials (RCTs) and observational studies that evaluated iptacopan for PNH. The primary efficacy outcomes were hemoglobin and lactate dehydrogenase (LDH) changes. A fixed-effects model was used for the meta-analysis. Six studies (three prospective cohorts, two RCTs, and one non-randomized trial) were included, comprising 197 patients. Iptacopan therapy significantly increased hemoglobin levels (mean differences (MD) = 12.98 g/L; 95% CI: 11.82-14.13; p < 0.0001) and decreased LDH (MD = -83.55 IU/L; 95% CI: -83.77 to -83.34; p < 0.0001). Subgroup analyses revealed more significant hemoglobin increases in European vs. Asian populations, studies with baseline Hb > 10 g/dL vs. < 10 g/dL, and studies lasting > 24 weeks vs. ≤ 24 weeks. LDH decreases were more pronounced in studies with baseline LDH > 500 IU/L vs. < 500 IU/L. The incidence of adverse events ranged from 66% to 90%, with the most common being headache, nasopharyngitis, and diarrhea. Serious adverse events occurred in 0-20% of patients across studies. Only one patient withdrew because adverse effects were reported across all studies. Preliminary data support iptacopan's effectiveness in improving hemoglobin levels and lowering hemolysis in PNH, both as a monotherapy and in combination with usual treatment. The safety profile appears to be excellent, with a minimal incidence of major adverse events and treatment discontinuation. Further studies are needed to validate the effectiveness and safety of larger, longer-term trials. Iptacopan is a viable oral therapy option for PNH.

## Introduction and background

Paroxysmal nocturnal hemoglobinuria (PNH) is a scarce and fatal blood condition characterized by complement-mediated intravascular hemolysis. It affects approximately 1-1.5 million people worldwide [1,2]. This life-threatening illness causes persistent hemolytic anemia, a high risk of thrombosis, and bone marrow failure. Mutations in the phosphatidylinositol glycan class A (PIGA) gene in hematopoietic stem cells induce PNH by preventing the production of protective proteins in red blood cells. As a result, these unprotected cells are left open to assault by the complement system, a critical component of the immune response that leads to red cell death when dysregulated [3,4].

The current standard of therapy comprises C5 complement protein inhibitors, such as eculizumab and ravulizumab. These medications significantly improve patient outcomes by lowering hemolysis and the need for transfusions; however, they are not without risks. Infusions are necessary for the rest of one's life, and many people find the expenses prohibitively expensive. Despite these advances, many patients continue to experience anemia and rely on transfusions, suggesting that additional complement-driven destruction occurs beyond the inhibition of C5 [5-7].

Iptacopan, a novel, orally administered targeted factor B inhibitor, is a promising development. This medicine showed promise in early studies by successfully lowering hemolysis and increasing hemoglobin levels, with lasting benefits, even without eculizumab [8]. Iptacopan inhibits factor B, which hinders the synthesis of C3 convertase and the subsequent assembly of the membrane assault complex, possibly resulting in more comprehensive complement suppression than eculizumab. Iptacopan's oral administration represents a substantial step toward more patient-friendly PNH care, indicating a less demanding and more comprehensive approach to illness control. This may modify the ordinary course of PNH and give patients hope for a more successful treatment plan [8,9].

The position of iptacopan in the PNH therapy landscape has been strengthened by phase 1 and 2 clinical studies investigating its effectiveness and safety. The data from these studies indicate that iptacopan is a revolutionary agent in PNH care, presenting an alternative to costly and intrusive therapies while meeting the unmet need for complete complement inhibition and enhanced quality of life (QOL) for patients with PNH [7,9]. This systematic review aimed to consolidate the available information on the effectiveness and safety of iptacopan in patients with PNH. However, information on the efficacy and safety of iptacopan is needed to establish its potential for significant improvement in PNH care. The findings are noteworthy because iptacopan may provide patients with a more effective, convenient, and accessible alternative therapy for this uncommon but dangerous blood condition.

## Review

Methodology

Study Design

This systematic review was conducted according to the Preferred Reporting Items for Systematic Reviews and Meta-Analyses (PRISMA) guidelines.

Data Sources and Search Strategies

A comprehensive literature search was performed using Medline, Embase, PubMed, and Cochrane Central Register of Controlled Trials. The search strategy combined the following Medical Subject Headings (MeSH) terms and keywords: "iptacopan," "LNP023," "factor B inhibitor," "PNH," "paroxysmal nocturnal hemoglobinuria," "complement-mediated hemolysis," and other relevant synonyms. Two investigators independently screened the retrieved studies against the predetermined eligibility criteria. Randomized controlled trials (RCTs) and observational studies assessing iptacopan for PNH treatment were included without language limitations. Two investigators independently extracted data on study characteristics, patient demographics, iptacopan dosing, efficacy outcomes, such as transfusion requirements and hemolysis, and safety outcomes, such as adverse events.

Inclusion Criteria

Participants: Patients diagnosed with PNH, confirmed by flow cytometry, demonstrating PNH clones. There were no restrictions regarding age, sex, or disease severity.

Interventions: Iptacopan monotherapy or combination therapy. Dose, route, frequency, and duration.

Comparators: Placebo, standard of care, or active comparator.

Outcomes: Efficacy outcomes, including hemoglobin levels, transfusion requirements, lactate dehydrogenase (LDH) levels, and QOL. The safety outcomes included adverse events and withdrawals due to adverse events.

Study design: RCTs, non-randomized controlled trials, prospective and retrospective observational cohort studies, and case-control studies.

Exclusion Criteria

Reviews, editorials, opinion pieces, and letters to the editor; studies that did not report iptacopan clinical efficacy or safety data; studies in which iptacopan was not specified or could not be isolated from combination therapies; and duplicate publications reporting the same patient population.

Quality Assessment

The risk of bias was evaluated using Cochrane's tool for randomized trials and the Newcastle-Ottawa scale (NOS) for observational studies. A meta-analysis was performed where feasible to synthesize the efficacy and safety results quantitatively.

Statistical Analysis

Mean differences (MD) were calculated for serum levels of hemoglobin and LDH before and after Iptacopan therapy. A fixed-effects model with the generic inverse variance method was used to calculate the pooled effect size. The results obtained from the pooled studies were demonstrated in forest plots, and a funnel plot was formed for the mean change in serum Hb levels to assess publication bias. The Higgins I square test was used to evaluate heterogeneity levels (low (<25%), moderate (25-75%), and high (>75%)) [10]. The analysis was deemed significant when the p-value was less than 0.05. All statistical analyses were performed using Review Manager (RevMan, version 5.4; Cochrane Collaboration, London, UK).

Methods for Exploring Heterogeneity

To explore the effect of clinical heterogeneity between the studies on meta-analysis outcome, subgroup analyses were performed based on the region for conducting the original research (Europe, Asia), age (<40 years, >40 years, and not mentioned), study design (RCTs, prospective studies, or non-RCT), duration of treatment (under 24 weeks, 24 weeks, and over 24 weeks), baseline Hb levels (< 10 g/dL and > 10 g/dL), baseline LDH levels (< 500 IU/L and > 500 IU/L), and mean baseline transfusion requirement (< 10, > 10, and unknown). Sensitivity analysis was performed to assess the contribution of each study to the pooled estimate by excluding individual trials one at a time and recalculating the pooled estimate for the remaining studies (leave-one-out meta-analysis) [11].

Results

Search Results

A flowchart illustrating the study selection is shown in Figure 1. Our search identified 571 records. These included 483 duplicate articles removed, leaving 88 unique articles for screening by title and abstract. Of the 136 articles screened, 69 were excluded because they did not meet the eligibility criteria, and two were not retrieved. The remaining 17 full-text articles were reviewed for more detailed evaluation, and 11 articles were excluded because eight did not report on the relevant drug iptacopan and three did not report on the appropriate study group. Finally, six studies were included in our meta-analysis.

**Figure 1:** PRISMA flowchart. PRISMA: Preferred Reporting Items for Systematic Reviews and Meta-Analyses

Study characteristics

Six eligible studies, three of which were prospective cohort studies [12-14], two of them being RCTs [15,16], and one was a non-randomized controlled trial [17], were included in the meta-analysis. The baseline and critical characteristics of the included studies are shown in Table 1. All of them were multi-center studies with a duration of iptacopan therapy ranging from 13 to 104 weeks.

**Table 1:** Baseline characteristics. LDH: Lactate dehydrogenase; IU/L: International units per liter.; g/L: Grams per liter; SD: Standard deviation; RCT: Randomized controlled trial; N/A: Not available

Study Name (Year of Publication)	Study Design	Country of Study	Sample Size (n)	Gender (n)		Mean Age (years)	Baseline Hemoglobin(g/L)	Baseline LDH (IU/L)	Transfusion Requirements at Baseline (n) Mean±SD
				Males	Females				
Risitano et al. (2021) [12]	Prospective Cohort	Italy, France, Germany	10	7	3	44.4±15.6	97.6±10.5	539±263	14.3±11.9
Peffault de Latour et al. (2023) [13]	Prospective Cohort	France, Italy	40	N/A	N/A	N/A	10	420	N/A
Ando et al. (2023) [14]	Prospective Cohort	Japan	10	N/A	N/A	N/A	90.3	420	11.4±3.8
Risitano et al. (2023) [15]	RCT	Italy, France, Germany, UK, Japan etc	62	N/A	N/A	N/A	10	N/A	N/A
Peffault de Latour et al. (2022) [16]	RCT	France, Italy	62	19	43	51±10.00	8.9±0.7	269.1±70.1	3.1±2.6
Jang et al. (2022) [17]	Non-randomized Control Trial	Korea, Taiwan, Malaysia, Singapore	13	7	6	37.21±12.55	87.18±11.66	2097.8±822.8	6.0±5.7

Risk of bias assessment

For prospective cohort studies, we used the NOS [18]. Table 2 presents the quality assessment of these three cohort studies. One had a low risk of bias (NOS score: 7-9), while two had a moderate risk of bias (NOS score: 4-6).

**Table 2:** Quality assessment of cohort studies. * indicates that the criteria have been met; - indicates that the criteria have not been met. For 1–9: Individual criteria in the Newcastle-Ottawa scale for assessing the quality of non-randomized studies Score: Total score on the Newcastle-Ottawa scale (maximum possible score is 9).

Study	Selection				Comparability		Outcome			Score
	1	2	3	4	5	6	7	8	9	
Risitano et al. (2021) [12]	*	_	*	*	_	_	*	*	*	6
Peffault de Latour et al. (2023) [13]	*	_	*	*	_	_	*	*	_	6
Ando et al. (2023) [14]	*	*	*	*	_	_	*	*	*	7

We used the NOS scale with some adaptations for the two RCTs and one non-RCT, as shown in Table 3. Two studies had a low risk of bias (NOS score: 5-7), and one study had a high risk of bias (NOS score: 0-4).

**Table 3:** Quality assessment of the controlled trials. * indicates that the criteria have been met; - indicates that the criteria have not been met. For 1–7: Individual criteria in the modified Jadad scale for assessing the quality of randomized controlled trials Score: Total score on the modified Jadad scale (maximum possible score is 7).

Study	Selection		Comparability		Outcome			Score
	1	2	3	4	5	6	7	
Risitano et al. (2023) [15]	*	*	_	_	*	*	*	5
Peffault de Latour et al. (2022) [16]	*	*	_	_	*	*	_	4
Jang et al. (2022) [17]	*	*	_	_	*	*	*	5

Evaluation of efficacy outcomes

Mean Change in the Hemoglobin Level

Our meta-analysis demonstrated that serum hemoglobin levels were significantly increased in patients after iptacopan therapy (MD = 12.98; 95% CI: 11.82, 14.13, p < 0.0001), as demonstrated in Figure 2. Sensitivity analysis was performed using the leave-one-out method to determine the primary outcome of the mean change in serum Hb levels. This sensitivity analysis showed no significant change in the pooled results after removing one of the studies.

**Figure 2:** Forest plot for the mean change in Hb levels. References: [12-17]

Mean Change in LDH Levels

The serum LDH levels were markedly decreased in patients after iptacopan therapy (MD = -83.55; 95% CI: -83.34, -83.77, p < 0.0001), as demonstrated in Figure 3.

**Figure 3:** Forest plot of the mean change in LDH levels. References: [12-14,17]

Subgroup analysis

Subgroup analyses were performed to explore the observed heterogeneity. Subgroup analyses were performed based on the region in which the original study was conducted (Europe, Asia), age (<40 years and >40 years), study design (RCTs, prospective studies, or non-RCT), duration of treatment (under 24 weeks, 24 weeks, and over 24 weeks), baseline Hb levels (< 10 g/dL and > 10 g/dL), baseline LDH levels (< 500 IU/L and > 500 IU/L), and mean baseline transfusion requirement (< 10, > 10, and unknown).

Subgrouping by Region

Sub-group analysis based on the region of the studies demonstrated that the mean change in serum Hb levels before and after therapy was significantly higher in European individuals than in the Asian population (Figure 4).

**Figure 4:** Subgrouping by region. References: [12-17]

Subgrouping by Age

Studies with a mean age of < 40 years showed a significantly more significant mean change in serum Hb levels before and after therapy compared to those with a mean age of > 40 years and those with an age not mentioned. However, the mean change in serum Hb levels before and after therapy was similar for studies with a mean age greater than 40 years and studies with age not mentioned (Figure 5).

**Figure 5:** Subgrouping by age. References: [12-17]

Subgrouping by Study Design

The mean change in serum Hb levels before and after therapy was significantly higher in prospective studies and non-RCTs than in RCTs (Figure 6).

**Figure 6:** Subgrouping by study design. References: [12-17]

Subgrouping by Duration of Treatment

The mean change in serum Hb levels before vs. after therapy was significantly higher in the study with a duration of treatment over 24 weeks compared to studies with a duration of therapy either less than or equal to 24 weeks (Figure 7).

**Figure 7:** Subgrouping by duration of treatment. References: [12-17]

Subgrouping According to Baseline Hemoglobin Levels

Our meta-analysis found that the mean change in serum Hb levels before vs after therapy was significantly higher in the studies with baseline Hb over 10 g/dL compared to studies with baseline Hb under 10 g/dL (Figure 8).

**Figure 8:** Subgrouping according to baseline hemoglobin levels. References: [12-17]

Subgrouping by Baseline LDH Levels

Our meta-analysis also found that the mean change in serum LDH levels before vs. after therapy was significantly higher in studies with baseline LDH > 500 IU/L than in studies with baseline LDH < 500 IU/L (Figure 9).

**Figure 9:** Subgrouping by baseline LDH levels. References: [12-14,17]

Subgrouping by Mean Baseline Transfusion Requirement

Finally, we found that the mean change in serum Hb levels before vs. after therapy was similar in the studies with mean baseline transfusion requirements under and over 10. Still, it was higher in the studies with unknown mean baseline transfusion requirements (Figure 10).

**Figure 10:** Subgrouping by the mean baseline transfusion requirement. References: [12-17]

Safety outcomes

Table 4 shows the incidence and incidence rates of adverse effects, serious complications, and patient withdrawal. Four of the six studies reported data regarding safety outcomes, and the incidence rate of adverse effects ranged from 66% to 90%. However, the incidence rate of serious complications is quite low, ranging from 0% to 20%. Moreover, only one patient across all six studies reported withdrawal from the therapy.

**Table 4:** Safety outcomes. N/A: Not available

Study Name (Year of Publication)	Incidence Rate of Adverse Effects n (%)	Severe Adverse Effects n (%)	Withdrawal Rate n (%)
Risitano et al. (2021) [12]	9 (90%)	2 (20%)	0 (0%)
Peffault de Latour et al. (2023) [13]	N/A	N/A	0 (0%)
Ando et al. (2023) [14]	6 (66.7%)	0	0 (0%)
Risitano et al. (2023) [15]	N/A	2 (5.7%)	0 (0%)
Peffault de Latour et al. (2022) [16]	47 (76%)	0 (0%)	0 (0%)
Jang et al. (2022) [17]	9 (69.2%)	0 (0%)	1(7.7%)

Discussion

This systematic review and meta-analysis provide persuasive evidence that iptacopan, an oral factor B inhibitor, is effective and safe for treating PNH. Our data showed considerable improvements in key hematological parameters and a favorable safety profile, indicating that iptacopan might be a potential step in PNH therapy.

The meta-analysis found a substantial increase in hemoglobin levels after iptacopan treatment (MD = 12.98 g/L; 95% CI: 11.82-14.13; p < 0.0001). This improvement is clinically significant and compares favorably with the outcomes of the existing standard-of-care therapies. For example, Hillmen et al. found that, after 36 months of eculizumab therapy, there was an average increase in hemoglobin of 10 g/L [19]. Similarly, the TRIUMPH study with eculizumab demonstrated a median hemoglobin rise of 5.5 g/L after 26 weeks [20]. Our meta-analysis revealed that iptacopan may provide greater hemoglobin improvements, perhaps leading to fewer transfusions and a higher QOL in patients with PNH.

Subgroup studies have elucidated the efficacy of iptacopan in various patient demographics and treatment scenarios. European research demonstrated a more significant rise in hemoglobin levels than in Asian studies, which might be attributed to genetic or environmental variables affecting treatment response. This geographic variance has not been thoroughly examined in previous PNH research and merits additional inquiry. Studies with a mean age of less than 40 showed a dramatic increase in hemoglobin levels, indicating that younger patients may benefit more from iptacopan. This age-related impact is comparable with findings from other PNH therapies, such as eculizumab, in which younger age was associated with better results [21].

Our research showed a significant reduction in LDH levels after iptacopan administration (MD = -83.55 IU/L; 95% CI: -83.77 to -83.34; p < 0.0001). LDH is an essential measure of intravascular hemolysis in PNH, and its decrease implies the efficient control of complement-mediated red blood cell destruction. The degree of LDH decrease observed with iptacopan was equivalent to that observed with eculizumab and ravulizumab. A previous study demonstrated an 87% decrease in LDH levels with eculizumab after 26 weeks [20], and our meta-analysis revealed a comparable reduction with iptacopan. This shows that iptacopan might be as successful as existing hemolytic treatments.

The safety findings of the included trials were favorable, with adverse event rates ranging from 66% to 90%. This aligns with the safety profiles of other complement inhibitors used in PNH therapy. Notably, the incidence of major adverse events was modest, ranging from 0% to 20% across trials. This excellent safety profile is consistent with the long-term safety data for eculizumab, which revealed significant adverse events in 22% of patients after a median follow-up of 30 months [22]. The low withdrawal rate in our study (one patient across all studies) adds to the tolerability of iptacopan and compares well with withdrawal rates found with other PNH treatments.

Iptacopan's action as a factor B inhibitor has numerous potential benefits over other terminal complement inhibitors, such as eculizumab and ravulizumab. Oral delivery may enhance therapy adherence and QOL in patients, addressing a major shortcoming of existing intravenous medicines. Iptacopan targets factor B and inhibits both the alternative and traditional complement pathways earlier in the cascade, potentially offering more extensive protection against hemolysis. This proximal inhibition may help address extravascular hemolysis, which can occur in individuals treated with C5 inhibitors. Risitano et al. discovered that up to 35% of eculizumab-treated individuals exhibited chronic extravascular hemolysis [23]. Our findings imply that iptacopan may solve this problem, but direct comparison studies are required to corroborate this notion.

Some of the studies in our study found that iptacopan therapy increased the size of the PNH red blood cell clones. This behavior, observed with various complement inhibitors, shows that PNH erythrocytes are well-protected and may contribute to long-term hematological responses. Kelly et al. found comparable results with eculizumab, reporting a median increase in PNH granulocyte clone size from 68.1% at baseline to 92.7% after 36 months of therapy [24]. Our findings showed that iptacopan might similarly affect PNH clone dynamics.

Limitations of this review and meta-analysis

Although our meta-analysis provided helpful information, some limitations should be addressed. Some analyses revealed significant heterogeneity, possibly due to research design variations, patient groups, and treatment procedures. Most of the included trials had very short follow-up periods, emphasizing the necessity for longer-term research to examine the durability of response and long-term safety of iptacopan. Furthermore, although our findings imply that iptacopan is equally or more effective than existing therapies, head-to-head trials comparing it to eculizumab or ravulizumab are required to establish its role in PNH care conclusively.

## Conclusions

This systematic review and meta-analysis prove that iptacopan is effective and safe for treating PNH. The considerable increase in hemoglobin levels decreased LDH, and the favorable safety profile offers iptacopan as a promising step in PNH therapy. Its oral delivery and distinct modes of action provide potential benefits over the current treatments. As research in this sector progresses, iptacopan may represent a paradigm change in PNH therapy, providing patients with a more convenient, effective, and well-tolerated alternative. Further research, particularly long-term follow-up and head-to-head comparisons with known medications, will be critical to determine the best place for iptacopan in the PNH therapy landscape.
